The article "A Prediction Model for Cognitive Impairment Risk in Colorectal Cancer after Chemotherapy Treatment" was retracted in 2024. Reasons: signs of a paper mill; suspected computer-generated content; unreliable results or conclusions; concerns about the results or conclusions.

# A Prediction Model for Cognitive Impairment Risk in Colorectal Cancer after Chemotherapy Treatment

**DOI:** 10.1155/2021/6666453

**Published:** 2021-02-20

**Authors:** Shu-Ping Zhou, Su-Ding Fei, Hui-Hui Han, Jing-Jing Li, Shuang Yang, Chun-Yang Zhao

**Affiliations:** Ningbo College of Health Sciences, No. 51, Xuefu Road, Yinzhou, Ningbo 315100, China

## Abstract

**Background:**

A prediction model can be developed to predict the risk of cancer-related cognitive impairment in colorectal cancer patients after chemotherapy.

**Methods:**

A regression analysis was performed on 386 colorectal cancer patients who had undergone chemotherapy. Three prediction models (random forest, logistic regression, and support vector machine models) were constructed using collected clinical and pathological data of the patients. Calibration and ROC curves and *C*-indexes were used to evaluate the selected models. A decision curve analysis (DCA) was used to determine the clinical utility of the line graph.

**Results:**

Three prediction models including a random forest, a logistic regression, and a support vector machine were constructed. The logistic regression model had the strongest predictive power with an area under the curve (AUC) of 0.799. Age, BMI, colostomy, complications, CRA, depression, diabetes, QLQ-C30 score, exercise, hypercholesterolemia, diet, marital status, education level, and pathological stage were included in the nomogram. The *C*-index (0.826) and calibration curve showed that the nomogram had good predictive ability and the DCA curves indicated that the model had strong clinical utility.

**Conclusions:**

A prediction model with good predictive ability and practical clinical value can be developed for predicting the risk of cognitive impairment in colorectal cancer after chemotherapy.

## 1. Introduction

Chemotherapy is a common complementary treatment for colorectal cancer. Cancer-related cognitive impairment (CRCI) occurs in cancer patients after chemotherapy [1–5].

The new treatment prolongs the life expectancy of cancer patients while it increases the incidence of CRCI. The National Cancer Institute (NCI) has indicated that CRCI should be thoroughly studied. CRCI has a substantial impact on the postoperative quality of life and the overall prognosis of patients [6, 7]. CRCI makes daily life and rehabilitation care difficult for cancer patients, leading to a reduced quality of life and a shorter life span [8, 9]. Therefore, it is important to explore the potential risk factors associated with the development of CRCI in colon cancer patients after chemotherapy. The knowledge of these potential risk factors can help to improve the overall prognosis of patients.

The article "A Prediction Model for Cognitive Impairment Risk in Colorectal Cancer after Chemotherapy Treatment" was retracted in 2024. Reasons: signs of a paper mill; suspected computer-generated content; unreliable results or conclusions; concerns about the results or conclusions.

The development of cognitive impairment in cancer patients is linked to various psychosocial or tumor-related factors [10]. However, there are no systematic assessment tools to predict the risk for CRCI complications in colon cancer patients after chemotherapy [11]. CRCI risk prediction is now possible because of the advancements in computer science and technology [12, 13]. A validated model can be developed to predict the CRCI risk in colorectal patients after chemotherapy. This is based on the existing clinical and epidemiological characteristics of patients who developed cognitive impairment after chemotherapy.

In this study, a predictive model was developed to predict the CRCI risk in colorectal cancer patients after chemotherapy to improve life quality. This model provides a clinical basis for individualized treatment options, especially for individuals at high CRCI risk. In conclusion, this study provides new ideas for improving the quality of life of colorectal cancer patients.

## 2. Materials and Methods

### 2.1. Patients

Data was collected from 386 patients who underwent surgery and postoperative chemotherapy between June 2016 and August 2020 at Ningbo Medical Center Lihuili Eastern Hospital. A retrospective analysis was then performed, and further questionnaires and follow-ups were conducted using telephone appointments and community follow-ups. The ethics committee of the hospital approved this study, and informed consent was obtained from patients or their families. Inclusion criteria were (1) postoperative pathologically confirmed diagnosis of colon or rectal cancer, (2) no history of other tumors or treatment, (3) no history of psychiatric drug use, (4) chemotherapy treatment, and (5) no organ failure occurrence. Exclusion criteria were (1) refusal to participate, (2) death during the study, (3) inadequate clinical or pathological information, (4) fever or infection of unknown origin, (5) metastatic tumors, and (6) inconsistent medical history with follow-up information.

### 2.2. CRCI or Depression Diagnosis

Experienced neuropsychologists examined the cognitive function using the Mini-Mental State Examination (MMSE) described in previous studies [14, 15]. The MMSE cut-off point for CRCI was similar to those in previous studies [16, 17]. An experienced psychiatrist assessed the depression diagnosis using the HAMD-17 (with good internal consistency and validity) [18, 19]. Depression diagnosis was made when HAMD‐17 ≥ 8, and its total score was between 0 and 54 [20, 21].

### 2.3. Patient and Clinical Statistical Characteristics

Clinical information (clinicopathological stage, tumor site origin, colostomy, basal heart rate, history of hypertension and diabetes mellitus, tumor-related anemia, and treatment complications) was collected and confirmed from the patient's medical history and follow-up survey one year after treatment. Patient demographic information including age, gender, height, weight, grip strength, smoking history, education level, marital status, alcohol consumption history, dietary preferences, and exercise frequency was also collected. The anemia status was evaluated using the WHO and American Cancer Institute (NCI) anemia grading criteria. Patients were diagnosed with CRA when their hemoglobin (Hb) was <120 g/L in men and <110 g/L in women.

The article "A Prediction Model for Cognitive Impairment Risk in Colorectal Cancer after Chemotherapy Treatment" was retracted in 2024. Reasons: signs of a paper mill; suspected computer-generated content; unreliable results or conclusions; concerns about the results or conclusions.

### 2.4. Rating Scale Collection

The Pittsburgh Sleep Quality Index (PSQI) with a Cronbach factor of 0.805 was used to assess the quality of a patient's sleep [22, 23]. The PSQI scores between 0 and 21 with higher scores indicate poor sleep quality. The Social Impact Scale including social exclusion, economic discrimination, inherent shame, and social isolation measures the patient's stigma [24]. The Chinese EORTC QLQ-C30 consists of 30 items divided into 15 sections. The scale scores range between 30 and 126. The higher the score, the poorer the patient's quality of life. The Chinese EORTC QLQ-C30 had good reliability and validity [25].

### 2.5. Statistical Analysis

All statistical analyses were determined using the R software (version 3.5.3). Patients were randomly divided into the training and validation groups (group ratio 7 : 3), and three models were selected. The model with the strongest predictive power was selected by calculating their respective AUC values. The stochastic forest model was effective at high latitudes and could quantify the importance of each feature and balance errors in the unbalanced data [26]. Support vector machines were effective in feature selection and the removal of redundant features, especially when dealing with small data [27]. Multiple logistic regression models are common and were also included. LASSO analysis was incorporated for dimensional reduction to filter the most suitable predictors to prevent overfitting [28]. The aim of this step was to select the core variables. LASSO regression has more advantages than ridge regression in terms of variable selection. Therefore, we choose LASSO regression to filter the variables as reported in a previous study [29]. ROC curves were used for visualization of AUC values to assess the accuracy of the model [30]. For models with high AUC values, the calibration curve and *C*-index were used to assess their predictive power further [31, 32]. Finally, the DCA curve was used to assess the clinical applicability of the model [33]. A *p* value less than 0.05 was considered statistically significant. A one-way ANOVA or two-tailed *t*-test was used to determine the significance between groups.

The article "A Prediction Model for Cognitive Impairment Risk in Colorectal Cancer after Chemotherapy Treatment" was retracted in 2024. Reasons: signs of a paper mill; suspected computer-generated content; unreliable results or conclusions; concerns about the results or conclusions.

## 3. Result

### 3.1. Demographic and Clinical Characteristics

Figure 1 illustrates the study flow. Clinical information of 386 colorectal cancer patients (189 women and 269 men) after chemotherapy treatment followed up between December 2014 and June 2020 was assessed. Patients were grouped into either the normal group (*n* = 269) or the CRCI group (*n* = 117). The differences in demographic and clinical characteristics between the CRCI and non-CRCI patients are shown in Table 1. Age, BMI, depression, alcohol consumption history, exercise frequency, diabetes history, colostomy, primary tumor focus, comorbidities, and CRA occurrence were statistically different between the CRCI and normal groups (*p* > 0.05).

### 3.2. Predictive Model Selection and Predictor Screening

Patients were randomly divided into the training and validation groups (group ratio 7 : 3), as shown in Table 2. Three models were selected, and the model with the strongest predictive power was finally obtained by calculating their respective AUC values. The stochastic forest model was constructed using important values for each factor (Figure 2(a)). The random forest model had an AUC value of 0.73 indicating that its predictive power should be improved. Model overfitting occurs in machine learning. The least absolute shrinkage and selection operator (LASSO) was used to reduce the number of features further to prevent model overfitting. The LASSO method is not effective in providing the same predictors each time. In this study, 1000 random LASSO regression analyses were conducted. These predictors were sequentially included in the logistic model according to the number of occurrences of the predictor. The final results suggested that the model had the most effective predictive ability when 14 predictors were included (AUC = 0.799) (Figure 2(b)). Support vector machine (SVM) models were more effective in selecting relevant features and removing redundant features than linear analysis. SVM models were also used to construct predictive models (Figure 2(c)) and had the strongest predictive accuracy (AUC = 0.7719) with 13 predictive factors. In summary, the LASSO-based logistic prediction model has the strongest predictive power for the CRCI risk in colorectal cancer patients after chemotherapy.

### 3.3. Building Visual Predictive Models

A visual nomogram prediction model based on a logistic model was developed to predict the CRCI risk in colorectal cancer patients after chemotherapy (Figure 3, Table 3). Age, BMI, colostomy, complications, CRA, depression, diabetes, QLQ-C30 score, exercise, hypercholesterolemia, diet, marital status, education level, and pathological stage were the 14 predictive factors.

The article "A Prediction Model for Cognitive Impairment Risk in Colorectal Cancer after Chemotherapy Treatment" was retracted in 2024. Reasons: signs of a paper mill; suspected computer-generated content; unreliable results or conclusions; concerns about the results or conclusions.

### 3.4. Nomogram Prediction Model Validation

The nomogram calibration curves showed good concordance, indicating that the model can be used to predict CRCI risk in colorectal cancer patients after chemotherapy (Figure 4(a)). Furthermore, the *C*-index was high in both the training and test groups, scoring 0.826 (95% CI, 0.774-0.877), 0.734 (95% CI, 0.633-0.835), and 0.796 (95% CI, 0.750-0.842), respectively (Table 4). An AUC value of 0.796 was achieved in the overall sample, 0.826 in the training group, and 0.734 in the test group (Figure 4(b)).

### 3.5. Clinical Application Evaluation

The nomogram results are shown in Figure 5. Findings showed that the decision curve using the nomogram prediction model had better clinical decision-making. The DCA revealed that when the threshold probability of a patient and doctor is 0% and 78%, respectively, in the entire cohort, using this nomogram provides additional benefits as reported previously [34]. Therefore, the model can predict CRCI risk in colorectal cancer patients after chemotherapy at an early stage. This can promote early clinical intervention, thus supporting personalized postoperative cancer rehabilitation.

## 4. Discussion

In this study, a LASSO regression model was used to obtain the most dominant factors influencing prognosis. The LASSO regression model had the most effective predictive power when the number of major predictors was screened down from 28 to 14. The predictive factors included age, BMI, colostomy, complications, CRA, depression, diabetes, QLQ-C30 score, exercise, hypercholesterolemia, diet, marital status, education level, and pathological stage. A risk prediction model was developed using these predictors to predict CRCI occurrence in colorectal cancer patients after chemotherapy. The test group was used to further evaluate the predictive model, and it was found to have good predictive ability and excellent performance in clinical decision-making. Therefore, this model can predict CRCI risk in colorectal cancer patients after chemotherapy at an early stage. This can facilitate early clinical intervention, thus improving the long-term prognosis of colorectal cancer patients.

Cognitive impairment is a transitional state from normal aging to dementia with 80% having dementia after six years [35]. The onset of Alzheimer's disease can be delayed if patients are intervened in the early cognitive impairment stages [36]. Therefore, research is necessary for efficiently diagnosing early AD patients and identifying prodromal AD stages. Nomogram prediction models have been widely used for disease-related prognostic analysis. The analytical results are visualized, greatly increasing the prediction accuracy and making them more suitable for clinical decision-making [37]. A nomogram prediction model was used to predict CRCI risk in colorectal cancer patients after chemotherapy. Three models were selected, and a nomogram prediction model based on logistic analysis was finally obtained by calculating their respective AUC values. In conclusion, this study establishes and validates a predictive model for predicting CRCI risk in colorectal cancer patients after chemotherapy. Some predictors in this study are related to CRCI risk in cancer patients. Cancer and cognitive impairment often coexist in old age. The burden of cancer and its treatment can lead to cognitive impairment [11]. There is a significant correlation between age and CRCI occurrence. Studies have found that overweight and high BMI are associated with a reduced risk of cognitive impairment in Chinese elderly people [38, 39]. Diabetes has also been identified as a possible risk factor for CIRC [40]. Previous studies have identified hypercholesterolemia as a vascular risk marker for injury recognition, and it has also been incorporated into the CRCI risk prediction model [41]. Patients with familial hypercholesterolemia (who experience cognitive impairment between 14 and 40 years) tend to develop mild cognitive impairment at 50 years [42]. A recent meta-analysis suggested that physical activity improves cognition in patients with mild cognitive impairment or dementia [43]. Several studies have also identified the positive impact of the Mediterranean diet on patients with cognitive impairment [44]. Therefore, physical exercise and a balanced diet are essential for early cancer recovery. Patients with a higher level of education show better compliance and recognize the importance of a healthy lifestyle in their recovery. Therefore, clinical education improves patients' perceptions of the disease [45]. Intensive clinical education can reduce CRCI risk in patients.

The article "A Prediction Model for Cognitive Impairment Risk in Colorectal Cancer after Chemotherapy Treatment" was retracted in 2024. Reasons: signs of a paper mill; suspected computer-generated content; unreliable results or conclusions; concerns about the results or conclusions.

Colostomies are also associated with cognitive impairment. Many patients require a colostomy after colon surgery. However, a stoma can have a serious impact on a colon cancer patient's diet, quality of life, and physical and mental well-being [46]. Surgical injury and treatment-related complications are key risk factors for cognitive impairment. Systemic inflammatory response activation damages the central nervous system [47]. Colorectal cancer and disease-related treatments (surgery, chemotherapy, etc.) contribute to cancer-related anemia. Studies have demonstrated that chronic anemia causes cognitive impairment regardless of age, kidney function, and HbA1c levels [48].

A good marriage can prevent cognitive impairment but is easily overlooked. Older people who are divorced or widowed are vulnerable to symptoms associated with cognitive impairment [49]. Therefore, postchemotherapy cancer patients' mental health should be taken into account, helping them face their new life with a more positive and optimistic attitude and increase their awareness of the disease and treatment [50] The patient's family and friends should also provide social support, thus improving their psychological condition [51].

This nomogram prediction model provides a basis for further research on CRCI risk in colorectal cancer patients after chemotherapy. Moreover, cognitive impairment biomarkers, cognitive evaluation, demographic data, clinicopathological characteristics, positron emission tomography data, functional magnetic resonance imaging, cerebrospinal fluid examination, and other data components should be added to the multimodal database for future studies. With the increase of sample size, the model would be further optimized. Further multicenter research should be supplemented to expand cooperation. The sample size of the study data should be increased to obtain a more accurate and stable predictive model for CRCI risk. Finally, further application of this predictive model may need to be adapted to clinical reality. In summary, a new predictive model has been developed to predict CRCI risk in colorectal cancer patients after chemotherapy. The model suggests that advanced age, colostomy, postoperative complications, diabetes, hyperlipidemia, divorce status, lower education, and the later pathological stage could be the risk factors for CRCI in colorectal cancer patients after chemotherapy. This study suggests that a balanced diet, adequate physical activity, and well-controlled diabetes are essential for cognitive maintenance in elderly patients. Mental health during the patient's illness should also be taken into account. The patient's social identity also needs to be promoted to reduce the risk of depression and CRCI.

## 5. Conclusion

In conclusion, a predictive model with a high degree of accuracy can be developed and validated to predict the CRCI risk in colorectal cancer patients after chemotherapy. The model provides a clinical rationale for individualized treatment options by identifying individuals' CRCI risk. It also provides new ideas for improving the quality of life of colorectal cancer patients.

## Figures and Tables

**Figure 1:** Flow chart of the study population.

**Figure 2:** Predictive model selection and predictor screening. (a) The random forest model. The graph on the left shows the importance of each factor in the random forest model, and the ROC curve demonstrates the accuracy of the random forest model (AUC = 0.730). (b, c) LASSO analysis conducted 1000 times. The factors were included in the logistic regression model to obtain a pattern diagram of the AUC for the number of occurrences. The model with 14 predictors had good predictive power (AUC = 0.799). (d) A prediction model developed using the SVM method with the highest prediction accuracy when 13 predictive factors are included (AUC = 0.7719).

The article "A Prediction Model for Cognitive Impairment Risk in Colorectal Cancer after Chemotherapy Treatment" was retracted in 2024. Reasons: signs of a paper mill; suspected computer-generated content; unreliable results or conclusions; concerns about the results or conclusions.

**Figure 3:** Building visual predictive models. Nomogram prediction model for CRCI risk in colorectal cancer patients after chemotherapy. Note the 14 factors including age, BMI, colostomy, complications, CRA, depression, diabetes, QLQ-C30 score, exercise, hypercholesterolemia, diet, marital status, education level, and pathological stage.

**Figure 4:** Nomogram prediction model validation. (a) Calibration curve of a model for predicting CRCI risk in colorectal cancer patients after chemotherapy. The closer combination of the solid and dashed lines indicates better predictive power. The predictive power of the model is shown using the ROC curve. (b) The AUC values for the training group (red), the test group (blue), and the encore cohort (orange) were 0.826, 0.734, and 0.796, respectively.

**Figure 5:** Clinical application evaluation. The DCA curve for this predictive model shows the decision analysis for the encore cohort, the training set, and the validation set.

**Table 1:** Differences of demographic and clinical characteristics between patients with and without CRCI.

Variables	Normal	CRCI	*p* value
	(*n* = 269)	(*n* = 117)	
Age	63.30 ± 9.59	68.03 ± 10.44	≤0.001^∗∗^
BMI	25.76 ± 3.44	24.95 ± 3.04	0.029^∗^
Waist	87.47 ± 9.14	87.32 ± 9.74	0.883
Heart rate	72.78 ± 8.63	73.19 ± 9.72	0.693
Depression			≤0.001^∗∗^
No	177 (65.80)	55 (47.01)	
Yes	92 (34.20)	62 (52.99)	
Gender			0.088
Female	124 (46.10)	65 (55.56)	
Male	145 (53.90)	52 (44.44)	
Smoking history			0.137
No	192 (71.38)	92 (78.63)	
Yes	77 (28.62)	25 (21.37)	
Education level			0.68
Higher education	66 (24.54)	27 (23.08)	
Primary education or below	100 (37.17)	49 (41.88)	
Secondary education	103 (38.29)	41 (35.04)	
Marital status			0.242
Single or divorce	76 (28.25)	40 (34.18)	
Married	193 (71.75)	77 (65.82)	
Medical insurance			0.701
Commercial insurance payment	46 (17.10)	16 (13.68)	
Social security payments	205 (76.21)	93 (79.49)	
Self-paying	18 (6.69)	8 (6.84)	
Homeplace			0.573
Rural areas	93 (34.57)	37 (31.62)	
Urban areas	176 (65.43)	80 (68.38)	
Per capita monthly household income			0.194
2001-5000 yuan per month	133 (49.44)	60 (51.28)	
<2000 yuan per month	48 (17.84)	28 (23.93)	
>5000 yuan per month	88 (32.71)	29 (24.79)	
Drinking			0.012^∗^
No	196 (72.86)	99 (84.62)	
Yes	73 (27.14)	18 (15.38)	
Diet			0.397
Balanced diet	82 (30.48)	42 (35.90)	
Carnivorous	101 (37.55)	36 (30.77)	
Vegetarian	86 (31.97)	39 (33.33)	
Exercise			≤0.001^∗∗^
Less than 3 times a week	131 (48.70)	52 (44.44)	
More than 3 times a week	64 (23.79)	6 (5.13)	
No	74 (27.51)	59 (50.43)	
Hypertension			0.733
No	175 (65.06)	74 (63.25)	
Yes	94 (34.94)	43 (36.75)	
Diabetes			0.043^∗^
No	212 (78.81)	81 (69.23)	
Yes	57 (21.19)	36 (30.77)	
Hypercholesterolemia			0.758
No	154 (57.25)	65 (55.56)	
Yes	115 (42.75)	52 (44.44)	
Pathological stage			0.239
No	125 (46.47)	62 (52.99)	
Yes	144 (53.53)	55 (47.01)	
Colostomy			0.010^∗∗^
No	235 (87.36)	90 (76.92)	
Yes	34 (12.64)	27 (23.08)	
Tumor location			0.039^∗^
Left hemicolon	67 (24.91)	23 (19.66)	
Rectum	103 (38.29)	50 (42.74)	
Right hemicolon	70 (26.02)	21 (17.95)	
Transverse colon	29 (10.78)	23 (19.66)	
Complications			≤0.001^∗∗^
No	244 (90.71)	92 (78.63)	
Yes	25 (9.29)	25 (21.37)	
CRA			0.012^∗^
No	53 (19.70)	11 (9.40)	
Yes	216 (80.30)	106 (90.60)	
PSQI	6.65 ± 3.74	7.26 ± 3.22	0.107
Social Impact Scale	62.43 ± 8.25	62.41 ± 7.62	0.985
Total score QLQ-C30	56.67 ± 11.98	55.09 ± 11.98	0.235

The article "A Prediction Model for Cognitive Impairment Risk in Colorectal Cancer after Chemotherapy Treatment" was retracted in 2024. Reasons: signs of a paper mill; suspected computer-generated content; unreliable results or conclusions; concerns about the results or conclusions.

**Table 2:** Differences of demographic and clinical characteristics between the training and testing sets.

Variables	Entire cohort	Training set	Testing set	*p* value
	(*n* = 386)	(*n* = 114)	(*n* = 272)	
CRCI				
No	269 (69.69)	79 (69.30)	190 (69.85)	0.994
Yes	117 (30.31)	35 (30.70)	82 (30.15)	
Age	64.73 ± 10.8	63.78 ± 9.11	65.13 ± 10.45	0.23
Gender				0.051
Female	189 (48.96)	44 (38.60)	145 (53.31)	
Male	197 (51.04)	70 (61.40)	127 (46.69)	
BMI	25.52 ± 3.34	25.70 ± 3.43	25.44 ± 3.31	0.49
Waist	87.42 ± 9.31	87.13 ± 9.94	87.54 ± 9.05	0.692
Heart rate	72.90 ± 8.96	71.91 ± 9.08	73.32 ± 8.90	0.161
Smoking history				0.08
No	284 (73.58)	75 (65.79)	209 (76.84)	
Yes	102 (26.42)	39 (34.21)	63 (23.16)	
Education level				0.465
Higher education	93 (24.09)	29 (25.44)	64 (23.53)	
Primary education or below	149 (38.60)	36 (31.58)	113 (41.54)	
Secondary education	144 (37.31)	49 (42.98)	95 (34.93)	
Marital status				0.73
Single or divorce	116 (30.05)	31 (27.19)	85 (31.25)	
Married	270 (69.95)	83 (72.81)	187 (68.75)	
Medical insurance				0.444
Commercial insurance payment	62 (16.06)	17 (14.91)	45 (16.54)	
Social security payments	298 (77.20)	85 (74.56)	213 (78.31)	
Self-paying	26 (6.74)	12 (10.53)	14 (5.15)	
Homeplace				0.947
Rural areas	130 (33.68)	37 (32.46)	93 (34.19)	
Urban areas	256 (66.32)	77 (67.54)	179 (65.81)	
Per capita monthly household income				0.961
2001-5000 yuan per month	193 (50.00)	60 (52.63)	133 (48.90)	
<2000 yuan per month	76 (19.69)	20 (17.54)	56 (20.59)	
>5000 yuan per month	117 (30.31)	34 (29.82)	83 (30.51)	
Depression				0.945
No	232 (60.10)	70 (61.40)	162 (59.56)	
Yes	154 (39.90)	44 (38.60)	110 (40.44)	
Drinking				0.556
No	295 (76.42)	83 (72.81)	212 (77.94)	
Yes	91 (23.58)	31 (27.19)	60 (22.06)	
Diet				0.576
Balanced diet	124 (32.12)	37 (32.46)	87 (31.99)	
Carnivorous	137 (35.49)	34 (29.82)	103 (37.87)	
Vegetarian	125 (32.38)	43 (37.72)	82 (30.15)	
Exercise				0.27
Less than 3 times a week	183 (47.41)	44 (38.60)	139 (51.10)	
More than 3 times a week	70 (18.13)	23 (20.18)	47 (17.28)	
No	133 (34.46)	47 (41.23)	86 (31.62)	
Diabetes				0.507
No	293 (75.91)	91 (79.82)	202 (74.26)	
Yes	93 (24.09)	23 (20.18)	70 (25.74)	
Hypertension				0.992
No	249 (64.51)	73 (64.04)	176 (64.71)	
Yes	137 (35.49)	41 (35.96)	96 (35.29)	
Hypercholesterolemia				0.441
No	219 (56.74)	59 (51.75)	160 (58.82)	
Yes	167 (43.26)	55 (48.25)	112 (41.18)	
Pathological stage				0.771
No	187 (48.45)	52 (45.61)	135 (49.63)	
Yes	199 (51.55)	62 (54.39)	137 (50.37)	
Colostomy				0.953
No	325 (84.20)	97 (85.09)	228 (83.82)	
Yes	61 (15.80)	17 (14.91)	44 (16.18)	
CRA				0.649
No	64 (16.58)	22 (19.30)	42 (15.44)	
Yes	322 (83.42)	92 (80.70)	230 (84.56)	
Complications				0.655
No	336 (87.05)	102 (89.47)	234 (86.03)	
Yes	50 (12.95)	12 (10.53)	38 (13.97)	
Tumor location				1
Left hemicolon	90 (23.32)	27 (23.68)	63 (23.16)	
Rectum	153 (39.64)	44 (38.60)	109 (40.07)	
Right hemicolon	91 (23.58)	27 (23.68)	64 (23.53)	
Transverse colon	52 (13.47)	16 (14.04)	36 (13.24)	
PSQI	6.83 ± 3.60	6.65 ± 3.64	6.91 ± 3.58	0.514
Social Impact Scale	62.42 ± 8.06	63.61 ± 8.53	61.92 ± 7.81	0.06
Total score QLQ-C30	56.20 ± 11.98	55.61 ± 12.19	56.44 ± 11.91	0.533

The article "A Prediction Model for Cognitive Impairment Risk in Colorectal Cancer after Chemotherapy Treatment" was retracted in 2024. Reasons: signs of a paper mill; suspected computer-generated content; unreliable results or conclusions; concerns about the results or conclusions.

**Table 3:** Prediction factors for CRCI.

Variables	Prediction model			
	*β*	Odds ratio (95% CI)		*p* value
Intercept	-2.316	0.099 (0.003-2.904)		0.181
Age	0.061	1.063 (1.034-1.094)		≤0.001
BMI	-0.073	0.929 (0.857-1.005)		0.072
Colostomy (yes)	0.736	2.088 (1.026-4.262)		0.042
Complications (yes)	0.998	2.712 (1.273-5.838)		0.010
CRA (yes)	0.835	2.306 (1.108-5.182)		0.032
Depression (yes)	0.612	1.845 (1.026-3.34)		0.041
Diabetes (yes)	0.518	1.678 (0.92-3.054)		0.090
Total score QLQ-C30	-0.008	0.992 (0.969-1.016)		0.517
Exercise				
Less than 3 times a week	-1.012	0.363 (0.202-0.643)		≤0.001
More than 3 times a week	-3.019	0.049 (0.015-0.132)		≤0.001
Hypercholesterolemia (yes)	-0.640	0.527 (0.285-0.955)		0.038
Diet				
Balanced	-0.645	0.525 (0.268-1.015)		0.057
Carnivorous	-0.587	0.556 (0.265-1.148)		0.116
Marital status (single or divorce)	0.512	1.669 (0.933-3.044)		0.089
Education level				
Secondary education	-0.375	0.687 (0.374-1.25)		0.221
Higher education	-0.395	0.674 (0.336-1.331)		0.259
Pathological stage (stage I&II)	-0.354	0.702 (0.416-1.176)		0.180

Note: *β* is the regression coefficient.

**Table 4:** *C*-index of the nomogram prediction model.

Dataset group	*C*-index of the prediction model	
	*C*-index	The *C*-index (95% CI)
Training set	0.826	0.774-0.877
Validation set	0.734	0.633-0.835
Entire cohort	0.796	0.750-0.842

## Data Availability

The datasets generated and analyzed during the present study are available from the corresponding author on reasonable request.

## Abbreviations

CRA: Cancer-related anemia
CRCI: Cancer-related cognitive impairment
DCA: Decision curve analysis
LASSO: Least absolute shrinkage and selection operator
ROC: Receiver operating characteristic curve
HAMD-17: The 17-item HAMD
PCA: Principal component analysis
PSQI: Pittsburgh Sleep Quality Index
QLQ-C30: European Organization for Research and Treatment Cancer Quality of Life Department C30
SIS: Social Impact Scale
SVM: Support vector machine
SSRS: Social Support Rate Scale.
